# Anti-NF155 chronic inflammatory demyelinating polyradiculoneuropathy strongly associates to HLA-DRB15

**DOI:** 10.1186/s12974-017-0996-1

**Published:** 2017-11-16

**Authors:** Laura Martinez-Martinez, Ma. Cinta Lleixà, Gemma Boera-Carnicero, Andrea Cortese, Jérôme Devaux, Ana Siles, Yusuf Rajabally, Alicia Martinez-Piñeiro, Alejandra Carvajal, Julio Pardo, Emilien Delmont, Shahram Attarian, Jordi Diaz-Manera, Ilaria Callegari, Enrico Marchioni, Diego Franciotta, Luana Benedetti, Guiseppe Lauria, Oscar de la Calle Martin, Cándido Juárez, Isabel Illa, Luis Querol

**Affiliations:** 1 Immunology Department, Hospital de la Santa Creu i Sant Pau, Universitat Autònoma de Barcelona, Barcelona, Spain; 2 Neuromuscular Diseases Unit, Department of Neurology, Hospital de la Santa Creu i Sant Pau, Universitat Autònoma de Barcelona, Mas Casanovas 90, 08041 Barcelona, Spain; 3 Centro para la Investigación Biomédica en Red en Enfermedades Raras, CIBERER, Madrid, Spain; 4 IRCCS Foundation C. Mondino National Neurological Institute, Pavia, Italy; 5 MRC Centre for Neuromuscular Diseases, National Hospital for Neurology and Neurosurgery, UCL Institute of Neurology, Queen Square, London, UK; 6 Centre de Recherche en Neurobiologie et Neurophysiologie de Marseille - CRN2M, UMR 7286, CNRS, Aix-Marseille Université, Marseille, France; 7 Regional Neuromuscular Clinic, Queen Elizabeth Hospital, University Hospitals of Birmingham, Birmingham, UK; 8 Neurology Department, Hospital Germans Trias i Pujol, Universitat Autònoma de Barcelona, Badalona, Spain; 9 Department of Neurology, Hospital Virgen de las Nieves, Granada, Spain; 10 Department of Neurology, Hospital Clínico de Santiago, Santiago de Compostela, Spain; 11 Referral Center for ALS and Neuromuscular Diseases, Timone University Hospital, Aix-Marseille University, Marseille, France; 12 Neuroscience Consortium, Monza Policlinico and Pavia Mondino, University of Pavia, Pavia, Italy; 13 Department of Neuroscience, Rehabilitation, Ophthalmology, Genetics, Maternal and Child Health, University of Genova and IRCCS AOU San Martino-IST, Genoa, Italy; 14 Neuroalgology Unit, IRCCS Foundation “Carlo Besta” Neurological Institute, Milan, Italy; 15 Department of Biomedical and Clinical Sciences “Luigi Sacco”, University of Milan, Milan, Italy

**Keywords:** CIDP, Antibodies, NF155, HLA DRB1*15

## Abstract

**Background:**

The aim of the research is to study the human leukocyte antigen (HLA) class II allele frequencies in chronic inflammatory demyelinating polyradiculoneuropathy (CIDP) associated with anti-neurofascin 155 (NF155) antibodies.

**Methods:**

Thirteen anti-NF155+ and 35 anti-NF155 negative (anti-NF155neg) CIDP patients were included in a case-control study. The frequencies of the DRB1 HLA allele were analyzed in all patients while DQ frequencies were only studied in patients sharing the DRB1*15 allele. In silico HLA-peptide binding and NF155 antigenicity, predictions were performed to analyze overlap between presented peptides and antigenic regions.

**Results:**

DRB1*15 alleles (DRB1*15:01 and DRB1*15:02) were present in 10 out of 13 anti-NF155+ CIDP patients and in only 5 out of 35 anti-NF155neg CIDP patients (77 vs 14%; OR = 20, CI = 4.035 to 99.13). DRB1*15 alleles appeared also in significantly higher proportions in anti-NF155+ CIDP than in normal population (77 vs 17%; OR = 16.9, CI = 4.434 to 57.30). Seven anti-NF155+ CIDP patients (53%) and 5 anti-NF155neg CIDP patients had the DRB1*15:01 allele (OR = 7, *p* = 0.009), while 3 anti-NF155+ CIDP patients and none of the anti-NF155neg CIDP patients had the DRB1*15:02 allele (OR = 23.6, *p* = 0.016). In silico analysis of the NF155 peptides binding to DRB1*15 alleles showed significant overlap in the peptides presented by the 15:01 and 15:02 alleles, suggesting functional homology.

**Conclusions:**

DRB1*15 alleles are the first strong risk factor associated to a CIDP subset, providing additional evidence that anti-NF155+ CIDP patients constitute a differentiated disease within the CIDP syndrome.

**Electronic supplementary material:**

The online version of this article (10.1186/s12974-017-0996-1) contains supplementary material, which is available to authorized users.

## Background

Chronic inflammatory demyelinating polyradiculoneuropathy (CIDP) is a heterogeneous autoimmune disease affecting peripheral nerves. Diagnosis relies on clinical and electrophysiological criteria built to identify patients that may respond to immunomodulatory treatments [1]. The recent description of antibodies targeting proteins at node of Ranvier, such as contactin-1 (CNTN1) [2], neurofascin-155 (NF155) [3], contactin-associated protein 1 (CASPR1) [4], and nodal neurofascins [5], has revealed the existence of CIDP subsets with clinical features that associate specifically to each antibody. In the case of anti-NF155, patients show predominantly distal weakness, ataxia, and a low frequency tremor [3]. They respond to intravenous immunoglobulins (IVIg) less frequently than anti-NF155neg CIDP [6], and when resistant to conventional treatment, they may respond well to B cell depleting therapies [7]. Anti-NF155 antibodies are predominantly IgG4, an isotype unable to fix complement or activate inflammatory cells [6]. Interestingly, anti-NF155 CIDP patients show distinct pathological features that differ from those of typical CIDP patients, including lack of macrophage infiltrates and a selective loss of the transverse bands at the paranodal loops [8, 9]. Thus, the clinical, pathological, and electrophysiological diversity of CIDP disappears when patients are sub-classified according to specific autoantibodies.

There is no epidemiological, environmental, or genetic evidence that explains the appearance of anti-NF155 antibodies, and evidence for the existence of CIDP-specific risk factors is lacking, including genetic association studies. Human leukocyte antigen (HLA) loci are the group of genetic factors that has most frequently been associated with autoimmune diseases, including strong associations with other IgG4-mediated diseases [10–12]. Moreover, association of HLA genes with specific antigens can help discover the specific peptide sequence driving the immune response [10]. Considering the association of other IgG4-mediated diseases to HLA class II, we aimed our study to identify specific HLA class II alleles associated to anti-NF155 antibodies in CIDP.

## Methods

### Patients, samples, protocol approvals, and patient consents

Patients fulfilling EFNS/PNS diagnostic criteria for CIDP that were positive for anti-NF155 antibodies were included [13]. CIDP patients without detectable anti-NF155 or anti-contactin-1 autoantibodies (anti-NF155neg CIDP) were used as controls. Serum and DNA samples were obtained from CIDP patients, processed and frozen until needed.

### Anti-NF155 antibody detection and isotype analysis

Antibodies against NF155 were detected by immunocytochemistry over human NF155 transfected-HEK293, and ELISA was used for autoantibody isotype identification as previously described [3].

### HLA genotyping

Genomic DNA from the peripheral blood of 13 anti-NF155+ CIDP patients, and 35 CIDP patients without anti-NF155 antibodies (anti-NF155neg CIDP) was extracted following standard protocols. HLA-DRB1 and HLA-DQB1 genotypes were determined at the four-digit allele levels using DNA sequence analysis following manufacturers’ instructions for HLA-DRB1 (SBT Excellerator GenDx HLA-DRB1, GenDx, Utrecht, Netherlands) and SSP methodology for HLA-DQB1 (All Set Gold SSP, One Lambda, California, USA). HLA-DRB1*15 allele frequencies were calculated for anti-NF155+ CIDP and compared with their frequency in anti-NF155neg CIDP patients and normal Spanish population (Spain-Barcelona, 941 controls included) previously published and available at public databases (allefrequencies.net) [14].

### In silico HLA-peptide binding and NF155 antigenicity predictions

In silico assays to predict NF155 binding to specific DRB1 alleles were developed using the IEDB analysis resource consensus [15, 16] and ProPred [17] tools during April and May 2017. The human NF155 sequence (NP_001153803.1) was used to predict peptides binding with higher affinity to those HLA alleles associated with anti-NF155+ antibodies. Peptides that were predicted to bind to both DRB1*15:01 and DRB1*15:02 alleles were considered.

Additionally, the Kolaskar and Tongaonkar antigenicity scale was used to predict NF155 antigenic targets. This scale values physicochemical properties of amino acid residues and their frequencies to predict antigenic determinants on proteins [18]. Predicted antigenic targets were compared with the results of the HLA-peptide binding prediction analysis in search of overlap.

### Statistical analyses

Data were collected in a coded database. Fisher’s exact test, odds ratio, and confidence interval calculations were performed using the GraphPad Prism v5.0 package.

## Results

### Association of anti-NF155 antibodies with DRB1*15

Thirteen CIDP patients with anti-NF155 IgG4 antibodies and 35 anti-NF155neg CIDP patients were included in the study. In all anti-NF155+ patients, antibodies were predominantly of the IgG4 isotype. As previously described [6] anti-NF155+ patients were younger than anti-NF155neg CIDP (47 vs 61; *p* = 0.03, Mann-Whitney), but there were no differences in gender or ethnicity. Demographic features are detailed in Table 1.

**Table 1:** Basic demographic data. CIDP patients with (NF155+ CIDP) or without (anti-NF155neg CIDP) anti-NF155 IgG4 antibodies showed similar gender proportions. They differed in age, NF155+ CIDP being younger than anti-NF155neg CIDP

	NF155+ CIDP	ANTI-NF155neg CIDP	
Gender (male, %)	69%	57%	ns
Age (mean)	47	61	*p* = 0.03^*^
Ethnicity—Caucasian (%)	92%	97%	ns

ns: non-significant; * Mann-Whitney

DRB1*15 alleles were present in 10 out of 13 anti-NF155+ CIDP patients and in only 5 out of 35 anti-NF155neg CIDP patients (77 vs 14%; OR = 20, CI = 4.035 to 99.13). Proportion of DRB1*15 alleles was also significantly higher in anti-NF155+ CIDP than in normal population (77 vs 17%; OR = 16.9, CI = 4.434 to 57.30) (Fig 1a). Seven (53%) anti-NF155+ CIDP patients, 5 (14%) anti-NF155neg CIDP patients (OR = 7, CI = 1.651 to 29.68), and 132 (14%) controls had the DRB1*15:01 allele (OR = 7.15, CI = 2.366 to 21.61) (Fig 1b). Finally, three (23%) anti-NF155+ CIDP patients, none (0%) of the anti-NF155neg CIDP patients (OR = 23.6, CI = 1.129 to 496.2), and 23 (2%) controls (OR = 11.97, CI = 3.088 to 46.43) had the DRB1*15:02 allele (Fig 1c). HLA results are detailed in Table 2.

**Fig. 1:** DRB1*15 allele frequencies. DRB1*15 alleles were present in significantly higher proportion of anti-NF155+ CIDP patients than anti-NF155neg CIDP or healthy controls, either in combination (**a**) or when analyzing DRB1*15:01 (**b**) and DRB1*15:02 (**c**) separately

**Table 2:** Detailed HLA class II results including DRB1 alleles from all patients and DQB1 from DRB1*15 positive patients

CIDP type	ID	DRB1*	DRB1*	DQB1*	DQB1*
NF155	1.BIR	3:01	4:01	02:–	3:01
NF155	5.ES	1:02	10:01	5:01	5:01
NF155	1.MAR	3:01	13:02	2:01	6:04
NF155	ITA-39	1:02	15:01	05:–	6:02
NF155	3.ES	1:02	15:01	5:01	5:02
NF155	4.ES	1:02	15:01	5:01	6:03
NF155	29.ES	4:04	15:01	3:02	6:02
NF155	19.ES	8:01	15:01	4:02	6:02
NF155	26.ES	11:04	15:01	6:02	6:02
NF155	2.MAR	14:01	15:01	5:01	6:02
NF155	ITA-40	7:01	15:02	02:–	6:01
NF155	23.ES	11:01	15:02	3:01	6:01
NF155	ITA-41	15:02	15:02	05:–	05:–
Negative	2.ES	1:01	1:03		
Negative	ITA-12	1:01	3:01		
Negative	ITA-10	1:02	3:01		
Negative	10.ES	3:01	3:01		
Negative	6.ES	1:03	4:02		
Negative	ITA-7	3:01	4:06		
Negative	ITA-18	1:01	7:01		
Negative	7.ES	3:01	7:01		
Negative	11.ES	3:01	7:01		
Negative	ITA-16	3:01	8:01		
Negative	8.ES	3:01	11:01		
Negative	ITA-6	4:07	11:01		
Negative	17.ES	7:01	11:01		
Negative	21.ES	10:01	11:01		
Negative	12.ES	3:01	11:04		
Negative	13.ES	4:01	11:04		
Negative	ITA-44	7:01	12:01	02:–	3:01
Negative	9.ES	3:01	13:01		
Negative	20.ES	10:01	13:01		
Negative	ITA-8	11:04	13:01		
Negative	ITA-11	1:01	13:02		
Negative	ITA-1	11:03	13:02		
Negative	1.ES	1:01	13:03		
Negative	24.ES	11:03	13:03		
Negative	ITA-2	11:04	13:03		
Negative	18.ES	7:01	13:05		
Negative	15.ES	7:01	14:01		
Negative	14.ES	4:02	15:01	03:–	6:02
Negative	16.ES	7:01	15:01	02:–	6:02
Negative	22.ES	10:01	15:01	05:–	6:02
Negative	ITA-9	11:04	16:02		
Negative	25.ES	11:04	15:01	03:–	6:02
Negative	27.ES	13:01	15:01	6:02	6:02
Negative	28.ES	11:01/04	16:01		

DQB1*6 alleles strongly associate with DRB1*15 alleles due to linkage disequilibrium. In our cohort, of those patients with DRB1*15 alleles, DQB1*6 was found in 8 anti-NF155+ CIDP patients and in all anti-NF155neg CIDP (80 vs 100%, non-significant) suggesting that the drivers of the association are the DRB1*15 alleles.

No other HLA class II allele was associated with anti-NF155 antibodies in CIDP, and DRB1 frequencies of anti-NF155neg CIDP patients did not differ to those of the general population.

### Prediction of NF155 peptide binding to DRB1*15

In silico prediction of NF155 peptides binding with higher scores to DRB1*15 yielded a significant overlap between the ProPred and IEDB prediction methods (Additional file 1). Most of the top peptides predicted for the DRB1*15:01 allele were also predicted for the DRB1*15:02, probably reflecting the minor differences between both alleles. Interestingly, one of the top 10 predicted peptides with all methods was also predicted with the highest antigenicity using the Kolaskar and Tongaonkar antigenicity scale (Additional file 1).

## Discussion

Our study finds a strong association of DRB1*15 alleles with anti-NF155+ CIDP compared to anti-NF155neg CIDP and general population. Specifically, anti-NF155+ CIDP patients have a DRB1*15 allele 20 times more likely than anti-NF155neg CIDP patients. This finding represents the first strong association of a CIDP subset with a specific genetic background and opens a new field =of study to investigate the interactions of the antigen presenting B cells, the T cells, and the immunological environment leading to IgG4 anti-NF155 antibody production.

Association of specific HLA alleles with autoimmune diseases is one of the most frequent topics of research in translational immunology and is used in several diseases (Behçet disease, ankylosing spondylitis, and others) as a diagnostic biomarker. Recent studies have found strong associations of certain HLA alleles in diverse tissue-specific IgG4-mediated diseases, such as LGI1 encephalitis (DRB1*07:01–DQB1*02:02 haplotype) [10], anti-MusK myasthenia (DR14-DQ5 haplotype) [19], or anti-IgLON5 disease (DRB1*10:01-DQB1*05:01) [11]. Early studies in CIDP did not find any association with specific HLA alleles, including studies addressing specifically the DRB1 frequencies in chronic autoimmune neuropathies. Other studies describe a weak association of specific HLA class I alleles with CIDP in some populations [20]. Considering that the effector mechanism in anti-NF155+ CIDP is B cell mediated, we focused in HLA class II associations, instead of HLA class I. Also, although this study did not aim to study specifically the association of HLA class II with anti-NF155neg CIDP, we did not find any difference in class II allele frequencies compared to general population.

DRB1*15 was not present in three (out of 13) anti-NF155+ CIDP patients, suggesting that HLA DRB1*15 is a strong risk factor but probably not a necessary factor for the development of anti-NF155 antibodies. This agrees with results in other IgG4-mediated diseases in which the associated HLA alleles are not universally found in all patients but with odds ratios ranging 8 to 100 and frequencies ranging 50 to 90% of patients [10, 19]. The DRB1 alleles found in those three anti-NF155+ CIDP, but DRB1*15 negative patients were also present in controls at similar frequencies; it is unlikely that they influenced their anti-NF155 antibody development.

The two DRB1*15 alleles found in CIDP patients (DRB1*15:01 and DRB1*15:02) reach statistical significance for their association with anti-NF155 antibodies independently. However, it is likely that the association with two different DRB1*15 alleles is not influencing the underlying peptide presentation process. DRB1*15:01 and DRB1*15:02 only differ in one amino acid (codon 86). Moreover, in silico experiments predicted common peptides binding to both alleles, suggesting that probably the same (or a very similar) peptide of NF155 could be presented with similar efficiency in both DRB1*15 alleles.

A limitation of our study is that, due to the low frequency of the disease, patients from four different origins (Spain, France, Italy, and UK) were included, while the statistical analysis where performed with Spanish controls. HLA-DRB1*15 is found in 17% of Spanish population, 12% of North Italy population, 25% of Southern France population, and 20% of English population (www.allelefrequencies.net). Considering the country of origin of the anti-NF155+ CIDP (7 Spain, 3 Italy, 2 France, and 1 England), these differences would not change the fact that anti-NF155+ CIDP patients show very high frequencies of DRB1*15 alleles compared to control populations, regardless of the origin of the control population used as reference.

Interestingly, DRB1*15 is also associated with multifocal motor neuropathy [21], although anti-NF155 are absent in this disease [22]; DRB1*15:01 also associates with multiple sclerosis [23], in which some studies described antibodies against NF155 associating to specific MS subtypes [24]. In fact, anti-NF155 antibodies have been described in patients with combined central and peripheral demyelination, but these findings have not been replicated in independent cohorts [25, 26]. None of our patients presented with symptoms or signs in the neurological exam suggesting central demyelinating disease. Moreover, 9 out of 13 anti-NF155+ patients had, at least, a brain MRI available and none of them showed central demyelinating lesions. Although DRB1*15 alleles have also been associated to other autoimmune diseases, including the IgG4-mediated anti-PLA2R membranous nephropathy [27], the association of DRB1*15 with three different diseases (multiple sclerosis, multifocal motor neuropathy, and anti-NF155+ CIDP) in which myelinating cells (oligodendrocytes and Schwann cells) are targeted by immune system may suggest convergent pathophysiological mechanisms in which myelin antigen presentation with DRB1*15 HLA class II is central. Some reports suggest that Schwann cells express HLA-DR in their surface, particularly in inflammatory neuropathies [28], but whether DRB1*15 alleles are expressed more efficiently in myelinating cells in comparison with other DRB1 alleles has never been studied.

## Conclusions

DRB1*15 alleles strongly associate to anti-NF155+ CIDP providing genetic evidence to support the idea that the clinical, electrophysiological, pathological, and genetic heterogeneity of CIDP disappears when the disease is segregated according to highly specific biomarkers like anti-NF155 antibodies.

## Additional file

Additional file 1: This excel file is composed by five different tables. **Tables S1** and **S2** display all peptides that the IEDB tool predicted to bind to DRB1*15:01 and DRB1*15:02 alleles, respectively, ordered by predicted binding strenght. **Table S3.** displays the 10 peptides binding with highest scores to DRB1*15 alleles as calculated by the ProPred tool. **Table S4.** displays all NF155 peptides ordered by their calculated antigenicity according to the Kolaskar and Tongaonkar antigenicity scale. **Table S5.** displays a summary of the findings relating the antigenicity scale findings with HLA-peptide prediction results with both IEDB and ProPred methods. (XLS 893 kb)

## Abbreviations

CASPR1: Contactin-associated protein 1
CIDP: Chronic inflammatory demyelinating polyradiculoneuropathy
CNTN1: Contactin-1
HLA: Human leukocyte antigen
IVIG: Intravenous immunoglobulin
NF155: Neurofascin-155
